# Design of an Intervention and Education System for Children with Emotional Disorders Based on Semantic Analysis

**DOI:** 10.1155/2022/4833968

**Published:** 2022-08-29

**Authors:** Ruifang Yang, Yiqun Wang

**Affiliations:** ^1^Department of Humanities Management, Erdos Vocational College, Inner Mongolia 017000, China; ^2^Logistics College, Beijing Institute of Materials, Beijing 100000, China

## Abstract

In this paper, a semantic analysis approach to children's emotional disorder intervention and education is thoroughly analyzed and discussed, and a corresponding educational system is designed for application in real life. This paper acquires video data by deploying a common camera acquisition and transforms, annotates, frames, and processes the data with the help of feature engineering methods. In addition, this paper proposes a fine-grained action decomposition strategy to solve the problem of extreme imbalance in the dataset to improve the performance of the model and proposes an iterative sampling data fusion strategy, which aims to integrate and fuse data from multiple sources to make them more effective and further improve the robustness and generalization ability of the model. Since it is difficult for families to improve the emotional management skills of migrant children, and it is also difficult to obtain professional help and support from the community or schools, it is important to take advantage of the professional strengths of social work to provide professional support for migrant children and their families. From the perspective of theoretical research, most of the existing studies focus on individual migrant children and cannot give global guidance from the perspective of the family system. The comparison results show that T-SVR trained using data from all subjects outperforms the inductive method based on individual training of trainees, validating the effectiveness of the proposed adaptive emotion recognition model. Therefore, from the perspective of system integration, it is important to explore social work interventions to improve the emotional management skills of migrant children. The system network structure design is determined according to the actual situation; then from the system requirements, the system is abstracted with the help of UML entity-relationship diagram, and the database table design is completed; so far, the overall system can be divided into independent functional modules, and the boundaries of each module and the participating roles are gradually clarified, and the detailed design within each functional module is illustrated by UML timing diagram and class diagram to clarify the classes used. Finally, the system is tested end-to-end to verify whether the results of the view layer meet the design guidelines, whether the system modules work together properly, and whether the functional development meets the requirements.

## 1. Introduction

Emotional interaction cannot be separated from the technical means of artificial intelligence. For nearly two decades, artificial intelligence researchers have been trying to empower machines with cognitive abilities to recognize, interpret, and express emotions. By correlating, analyzing, and reconstructing data containing emotional information in different scenarios, artificial intelligence technology finally transforms the data into abstract thoughts that computers can understand, thus simulating human emotional cognition and decision-making processes [1]. In other words, the emotional interaction process uses the user's modal data to recognize the user's emotional state and uses the feedback information from the emotional recognition to model the emotion based on cognitive analysis and to guide the interaction behavior [2]. The product-related category involves the homepage management module, course management module, store management module, and shopping cart management module, which aims to provide richer design elements, more beautiful style and layout, and more structured and themed display effects. Therefore, the emotion recognition process and the emotion modeling process are the two most important steps of affective interaction. Emotion is not only an individual's psychological change but also a social phenomenon [3]. Emotion is integrated into an individual's daily life and runs through his or her development, and the ability of emotion recognition, emotion expression, and emotion regulation profoundly affects an individual's physical and mental health and the development of his or her social competence [4]. Depression is gradually becoming the second leading cause of death after cancer, and minors have become one of the key groups of depressed patients [5]. From the perspective of developmental stage theory, children already have the basic emotion experience and emotion regulation ability and are in an important period of emotion awareness management ability development, which is an important part of social competence and profoundly influences the psychological characteristics and behavior of individuals in later development [6].

Cognitive psychology considers the adolescent period to be extremely important, and with the development of neuroscience, the adolescent period is one of the key stages in the social and emotional development of individuals [7]. From adolescence to early adulthood, individuals are and will remain in a critical period of neurodevelopment for a long time, and this period is accompanied by dramatic changes in hormonal and emotional experiences [8]. As a result, many psychiatric disorders first appear in adolescence and early adulthood, with approximately half of them occurring between the ages of thirteen and eighteen, but many parents and other primary caregivers may consider adolescent emotional and behavioral problems to be “perfectly normal” and “common at this age” [9]. The more samples in the dataset, the smaller the interval. Typically, the initial value of the learning rate is set to 0.0003. However, many parents and other primary caregivers may believe that adolescents' emotional and behavioral problems are “normal” and “common at this age” and that clinical consultation rates are low [10]. Adolescent mental disorders are often overlooked at the clinical and public health levels [11]. However, research has found that psychiatric disorders in adolescence and early adulthood are fully capable of disrupting individuals' social role transitions, such as transitioning from student to workplace roles, establishing lifelong partnerships, and achieving economic independence. There is evidence that investing in anxiety and depression can have a significant financial return. Anxiety disorders are also among the most common psychiatric disorders in children and adolescents [12, 13].

Treatment of adolescents with anxiety disorders should consider the physical and developmental status of the adolescent, and a variety of treatments, including medication and psychotherapy, are commonly used. Pharmacological treatment includes western medicine and herbal medicine [14]. Western medicine such as sertraline plays an active role in reducing clinical symptoms of adolescent anxiety disorder patients [15]. Chinese medications such as liver detoxification capsules can reduce symptoms in adolescent patients with anxiety disorders [16]. Psychotherapy should be considered as the first choice in the treatment of children and adolescents with anxiety disorders [17]. When the Faster R-CNN + ResNet50 and Faster R-CNN + ResNet101 models are learned in a step-decay mode, the accuracy of the model increases more, and the performance of the model is better when it is finally stabilized. When symptoms of anxiety disorders are moderate to severe, or when dysfunction makes participation in psychotherapy difficult, or when psychotherapy is only partially responsive, pharmacological treatment is recommended, starting with a low dose, closely monitoring for adverse effects, and slowly increasing the dose according to treatment response and tolerability [18]. Psychotherapy may disregard the concomitant disorders of anxiety and can be a good treatment for anxiety itself [19]. Most adolescents with anxiety disorders have negative automatic thought patterns, and cognitive behavioral therapy is an extremely effective and widely used treatment for adolescents with anxiety disorders [20]. In addition, physical therapy such as hypnosis and suggestion therapy are also available [21]. If the clinical symptoms are severe and persist without relief from severe suicidal behavior, twitch-free electroconvulsive therapy can be used [22].

Young children are at a rapid stage of psychological and behavioral development and have a great deal of plasticity [23]. Once physical and psychological problems are detected in young children, it is easier to intervene to correct them, which not only ensures their overall physical and psychological development but also brings greater social effects [24]. Nobel Laureate Heckman has suggested that interventions in early childhood development can yield an input-output ratio of 1 : 17. Investing in early childhood development is one of the most rewarding investments in human capital. Poverty reduction through early childhood development interventions has long been a central global concern, and the President has officially stated in his report to the 19th National Congress that emphasis should be placed on early childhood development. Early intervention for early childhood behavior problems is an educational initiative that can yield large returns. Traditional monolithic application architectures struggle to deal with this kind of problem: each change requires redeployment of the entire system, long compilation and testing cycles, coupling of algorithms and application frameworks, and wholesale changes for local component updates.

## 2. Method

### 2.1. Semantic Analysis

After the work of unimodal feature extraction is completed, the effectiveness of sentiment recognition after the fusion process is often limited due to the different methods and focus of each unimodal sentiment feature extraction [25].

Some works treat data characterizing inconsistent sentiment semantics as outliers and use traditional methods for handling outliers to filter them [26]. These traditional methods measure the similarity of incoming features and treat data with less similarity as outliers. However, this calculation of similarity may incur great computational and time costs, limiting the real-time application in practical situations. In addition, the similarity computation between high-dimensional multimodal features can lead to the “curse of dimensionality” problem. In contrast, the use of embedding vectors can avoid the computation of too many dimensions and enable the processing of features with different dimensions [27]. The embedding vectors cover the relationship between modal features and the corresponding sentiment semantics and thus can indirectly measure the similarity between different modal features [28]. Therefore, this chapter proposes a multimodal feature processing method combined with sentiment semantic analysis, using complementary information between sentiment semantics and multimodal features, to reduce the effects of multimodal features such as redundancy and mutual exclusion and further improve the performance of sentiment recognition. If the online user completes the transition to the parent role, this function can be unlocked, which is the only difference between the online user and the parent in the function of this system. The correlation between modality and semantics in the potential embedding space is measured, and the features are further processed using logistic stee regression to implement a multimodal fusion approach with a soft attention mechanism [29].

Therefore, this chapter is aimed at extracting multimodal features related to affective semantics using the means of affective semantic analysis, which makes multimodal features characterize affective semantics consistently. To consider the sentiment information associated between the modalities, the influence of the remaining low-level descriptors that are not related to the sentiment semantics is ignored, as shown in Figure 1.

Some target detectors in real-time detection in HD video are designed for image detection in general, but lack understanding of the correlation between frames in behavioral analysis [30]. In this regard, this paper proposes an action recognition model with continuity and spatiotemporal characteristics, which is mainly used to complete action semantic analysis by exploring spatiotemporal correlation and continuity of action sequences. Here, this domain model is called an action semantic recognition model with continuity and spatiotemporal characteristics, i.e., action spatiotemporal model (STM), which is mainly used to understand and perceive the set of action sequences with continuity and spatiotemporal characteristics for semantic analysis in this paper [31].

Descriptive statistical analysis was used to derive the mean and standard deviation of parenting style, young children's verbal ability, and behavioral development to have the most basic and comprehensive understanding of parenting style, young children's verbal ability, and behavioral development [32]. A chi-square analysis was used to compare the differences in the detection rates of behavior problems among different age groups of toddlers to understand the development of behavior problems in toddlers. Gender differences in behavior problems were compared using independent samples *t*-tests to understand gender differences in behavior problems in young children [33]. On the one hand, under the supervision of parents, you can conduct online course learning, online assessment, view the curriculum, and check the learning progress in this system. Analysis of variance (ANOVA) was used to compare the differences in the level of speech development, father's parenting style, and mother's parenting style of toddlers at different ages to understand the differences in the level of speech development and parenting style of toddlers at different ages [34].

The correlations between parenting styles and toddlers' behavioral development, toddlers' speech development and behavioral development, and parents' parenting styles and toddlers' speech development were obtained by using inferential statistical analysis, and the predictive effects of parenting styles and toddlers' speech development on toddlers' behavioral development were obtained by using regression analysis on top of the correlations [35]. The results were used to draw conclusions and make corresponding educational suggestions.

The types of behaviors in different contexts are different, and the corresponding types of actions are different. When the performance of the algorithmic model needs to be improved, then the algorithmic model performs better in feature extraction, feature representation, and detection recognition [36]. Although the behavior types are diverse, the features possess characteristics such as abstraction and liability. Based on these characteristics, convolutional neural networks are good at multilayer feature representation of the target to represent the abstract semantic information of the data with higher-level features, thus obtaining better feature robustness. Therefore, the stronger the FE's deep mining ability to extract features, the better the STM model's ability to learn the features.

### 2.2. Emotional Disorder Intervention

Emotional expressiveness refers to the ability of children to express their emotional states to the outside world and others through verbal language, facial expressions, and physical body based on the recognition and understanding of their own emotions [37]. Education should be a practical activity based on psychology, philosophy, and other disciplines, and scientific educational suggestions should be based on the scientific conclusions of psychology. The ability to express emotions accurately and effectively not only regulates emotions to a certain extent but also helps individuals to have better social interactions. However, from the statistical analysis of this research study, the mean value of the study sample's emotion management ability was the lowest among the three dimensions, at 23.91 points, and the lowest score of the sample was only 9 points. It is evident that the students of this school have relatively low ability to express their emotions and cannot better express their emotions to the outside world.

The mean scores of female students in all three dimensions are higher than the mean scores of male students. In the dimension of emotion control, the greatest difference was found in the mean scores of students of different genders, with the mean score of 26.68 for girls and 24.63 for boys, followed by the mean scores of emotions understanding and emotion expression. Based on the differences in the means of the three dimensions, the emotional management ability of male students in this school is slightly lower than that of female students in comparison, as shown in Table 1.

The teacher's description shows that there are some differences in the performance of students of different genders in coping with emotional changes. On the one hand, girls in this school showed better motivation in expressing their emotions than boys and were able to take the initiative to express their emotional changes to teachers or others [38]. On the other hand, boys are more likely to engage in problematic behaviors such as arguing and fighting under the influence of negative emotions. This also confirms the gender difference in students' emotion management skills, meaning that girls at the school are better able to express and control their emotions than boys and are less likely to engage in problematic behaviors under the influence of negative emotions.

In terms of individual developmental characteristics, for students in their formative years, the level of emotion management skills should increase with their age as their behavioral and cognitive abilities improve. This hypothesis is corroborated by the results of existing research on preschoolers aged 3 to 6 years, which shows a trend of change in the emotion management skills of children at different ages [39]. Compared with boys, girls in this school can better express and control their emotions, and they are less likely to have problem behaviors under the influence of bad emotions. Therefore, to test this hypothesis by understanding the differences and trends in the levels of emotion management skills of students at different age groups in the school, the sample of students in grades 3 to 6 was selected based on grade levels.

The test of differences between children with and without anxiety disorders on the dimensions given by SCARED tells us that children with anxiety disorders scored significantly higher than children without anxiety disorders, both on the total score of anxiety disorders and the dimensions [40]. It can be hypothesized that children with nonanxiety disorders are more receptive to going to school, more comfortable with daily social activities with their teachers and classmates, more open to separation from close relationships, calmer when encountering other life events, and less anxious emotional and physiological reactions than children with anxiety disorders, as shown in Figure 2.

In the intervention for children with anxiety disorders, a “case study” approach was used. Considering the shortcomings of the “case study method” and the accuracy of the research design, a matched group design was introduced, in which the subjects were divided into two groups according to their gender, age, class, and scale scores to implement different treatments (with/without box-trial therapy intervention), thus minimizing the influence of irrelevant variables [41]. Accurate and effective emotional expression can not only regulate emotions to a certain extent but also help individuals achieve better social interactions. However, from the statistical analysis results of this survey, the mean of the emotional management ability of the research sample is the lowest of 23.91 points in the three dimensions. As for the examination of the effects of box court therapy, it cannot be collected by traditional quantitative methods, and much of the rich and detailed and valuable information was obtained during the intervention and the interaction between the researcher and the subjects, so a qualitative study combined with a quantitative study was mainly adopted to examine the effects comprehensively.

Firstly, empirical survey research is mainly used in the research on young children's behavior, and the research method is relatively single; secondly, most of the research on young children's behavior stands only from the perspective of young children's psychology and lacks the part of making systematic educational suggestions based on the conclusions after drawing relevant or predictive relationships; education should be a practical activity based on psychology, philosophy, and other disciplines, and scientific-educational suggestions should be more based on psychology [42]. Finally, research on early childhood behavior lacks dynamic understanding; early childhood is a period of rapid physical and mental development of individuals, so early childhood behavior research should be explored more from a developmental perspective, such as the relationship between family factors and early childhood behavior; although they are all preschool, different ages may have different sensitivities to family factors, which is a dynamic developmental process, but most research on early childhood behavior problems are static studies, mainly looking at early childhood as a whole and studying its influences, etc.

### 2.3. System

Microservices is a style of software architecture that is based on small functional blocks focused on a single responsibility and task and uses a modular approach to assemble large, complex applications, with the functional blocks communicating with each other using a language-independent set of APIs [43]. Microservices take business functions as the division unit and divide different functions into different services; each service is an independent application that can run separately, and each service is connected with a specific communication protocol to form a system together. When the system performance bottleneck only needs to expand the capacity of the corresponding service, without the need to modify the rest of the system, there is a low coupling between the functional modules, easy to update the system, and flexible allocation of resources. However, as a distributed software architecture, the practice of microservices also needs to address the following issues.

The main products of this educational institution are two types, namely, online courses and offline courses, as shown in Table 2. Psychotherapy does not consider the accompanying diseases of anxiety and has a good therapeutic effect on anxiety itself. The teaching contents and modes of online and offline courses are different. The offline courses are taught by the offline stores, which is a long time and stage teaching and requires the cooperation and supervision of the offline stores, parents, and students to ensure the teaching effect. Online courses belong to the headquarters of the institution and are an independent unit form of video teaching, by the user to determine the content of the course, after the purchase of self-study. Online courses are sold and used in this system, so we need to provide functions such as viewing, purchasing, paying, and online learning. Offline course sales and use are not related to this system, so this system will be used as a promotional channel to display them only.

This system needs to display the educational products and industrial layout of the institution to the public, including store information and course information. Since offline stores are managed by the institution's headquarters, the store information required by this system is managed and maintained by the institution's headquarters [44]. Similarly, since the institution's headquarters publish the syllabus of online courses and offline courses, and the special courses of offline stores are also approved by the institution's headquarters, the course information is also managed and maintained by the institution's headquarters. The system is responsible for organizing and summarizing all kinds of information and presenting it to users in a suitable form, to achieve effective information communication effect.

For example, the display of store information is to attract customers to the offline stores, so it can provide content more in line with users' needs through geographic location filtering, store detail description, store faculty display, store teaching content display, store class schedule display, store teaching results display, etc. Individuals with common mental disorders during adolescence are more difficult to participate in formal education, employment, and training; those with self-injurious behavior are at higher risk for later mental and substance use disorders, and those who use marijuana and other illicit substances have better overall life outcomes. And the course information display is to attract users to learn the course; users can choose the learning channel according to the type of course online purchase online course learning or go to offline stores to register members to participate in offline course learning.

For linkage function with offline stores, this system is mainly for online users; in addition to online users, it should also provide online + offline joint teaching services for offline store members. The teaching target of this educational institution is children aged 3-12 years old; because of their young age, they need parental supervision, so the offline store will provide the parental account and student account associated with this system for the newly registered members, so the students can study offline courses in the offline store on one hand, and on the other hand, they can study online courses, online assessment, check the schedule, and view the learning progress in this system under parental supervision [45]. The students' learning situation is recorded and managed by the offline stores, so the offline stores are responsible for maintaining this part of the data. Online assessment is a set of relatively independent and complex functions related to the store management system and headquarter management system, which is not very related to the main content of this topic, so we will not discuss it later, but only for understanding.

Users registered online in this system are collectively referred to as online users. Since registration activities are user actions, this system does not supervise them; i.e., this system is not responsible for controlling the actual age and actual identity (parent, child) of online registrants and provides the public service type functions of this system for such accounts uniformly. The online course learning included in the public service is independent modular independent learning, and the online user arranges the learning mode by himself/herself. For example, a parent (meaning the actual life parent identity, different from the parent role in this system) can register online in this system to become an online user, purchase the course online, and then instruct the child to use the account to learn online. Since the membership service is to manage and synchronize the learning of registered members in offline stores, and online users have nothing to do with offline stores, they cannot use the membership service (only the membership service provides the function of associated accounts); i.e., online users are independent and do not have associated accounts, as shown in Figure 3.

The basic functions of the system are the login and registration functions common to all users (online users, parents, students), which are part of the public services mentioned above. Users may forget their passwords when logging in, so a forgot password use case is extended after the login use case, and users may also need to log out after logging in, so a logout use case is extended (the extended use case is not necessarily executed).

The personal center function is intended for the parent role and online user role, which can use this function for personal account management. The personal center function can be divided into five functions: view personal information, modify personal information, student management, view the list of course favorites, and view purchased records. Depression is gradually becoming the second leading cause of human death after cancer, and minors have also become one of the key groups of people with depression. The student management function includes four subfunctions: view personal information of associated students, modify the password of associated students, view class schedule of associated students, and view assessment results of associated students, which is a membership service linked with offline stores as mentioned above and therefore cannot be used by online users. This function can be unlocked if the online user completes the conversion to the parent role, which is the only difference between the online user and the parent in terms of the functions of this system.

The student management function includes four subfunctions: viewing the personal information of the associated students, changing the password of the associated students, viewing the class schedule of the associated students, and viewing the assessment results of the associated students. This function is also the main difference between the parent role and the online user role because the online user is not registered in the offline store; there are no associated students and therefore cannot manage the student information. Similarly, personal information, class schedule, assessment results, and other data are uploaded and maintained by offline store staff through the store management system.

If a parent account is associated with more than one student account, it will be displayed as a list of students. After viewing the students' personal information, parents can change the password of the students' accounts, thus extending the use case of changing the password of the associated students. In addition, parents can view the class schedule of the associated students through the student management function, which is convenient for taking care of their children and supervising their children's learning, as well as viewing the assessment results of the associated students to check the learning results of the associated students at each stage.

## 3. Results

### 3.1. Semantic Analysis Results

Another optimization goal is to optimize the learning rate using hyperparameters. Considering the complexity and training cost of the model, this paper mainly uses two model architectures, Faster R-CNN + ResNet and SSD + ResNet, to design and conduct experiments, and the learning rate adjustment strategies involved are mainly the segmented constant decay learning rate adjustment strategy and the cosine decay learning rate adjustment strategy. To explore the impact of the segmented constant decay-based learning rate adjustment strategy on the model accuracy, two model architectures, Faster R-CNN + ResNet50 and Faster R-CNN + ResNet101, are chosen to design and conduct a series of ablation experiments in this paper. In the experiments, it is often necessary to consider the setting of parameter interval values. Such parameters can be moderately adjusted according to the size of the dataset, and the more samples of the dataset, the smaller the interval. In general, the initial value of the learning rate is set to 0.0003.

Figure 4 shows the model accuracy change curves for both Faster R-CNN + ResNet50 and Faster R-CNN + ResNet101 models with and without step decay at the same time as the number of iterations increases. Figure 4 shows the learning rate change curves of both models with and without step decay scenarios as the number of iterations increases. Combining the two graphs clearly shows that at the beginning of model training, the model follows an initial learning rate for training and learning, and then, there are two ways to learn: one is that the learning rate does not change and keeps a constant value for continuous learning, and the other is to adopt a certain strategy to keep learning and reasoning with step decay.

According to the trend change of the model accuracy curve, it can be concluded that the model with a certain strategy of learning with step decay will continue to reduce the learning rate as the number of iterations increases, which can further reduce the loss as much as possible through finer iterations and avoid convergence of the model to the saddle point or the minimal value point, to improve the accuracy of the model. In contrast, the model learned by step-free decay keeps a constant initial value and keeps reasoning, which is more likely to fall into the saddle point or the minima point, and once it falls into it, the model cannot escape from this “trap” and will eventually perform poorly. The emotional interaction process uses the user's modal data to realize the recognition of the user's emotional state and uses the feedback information of emotion recognition to carry out emotional modeling based on cognitive analysis and to guide the interaction behavior. It can be learned that the Faster R-CNN + ResNet50 and Faster R-CNN + ResNet101 models with step decay learning have a greater increase in model accuracy and better performance when the model is finally stabilized.

The reasons for this result are mainly reflected in two aspects: network structure and data characteristics. First, the network structure is deeper and more complex than MobileNet-v1 and Inception-v2, and the residual network ResNet is deeper and wider than the former. Generally, the more complex the structure of the feature extraction network, the better the feature extraction effect is, which can improve the accuracy of the detection task to some extent. In addition, ResNet101 is based on ResNet50 with the addition of the fourth layer of convolutional blocks, which makes the network deeper in layers and therefore will perform better in deep mining and extraction of semantic features.

Another perspective, the structure of the detector focuses on the accuracy and recognition speed of the detector. In general, for a detection task, the detector is required to maintain semantic information while maintaining sufficiently accurate location information to obtain good feature alignment and good localization results. Compared with the two-stage-based detector Faster R-CNN, SSD detects and identifies the target in the image directly by one run, which does not perform particularly well in terms of detection accuracy and cannot meet the practical requirements.

### 3.2. System Performance

The system design is positioned as a portal, mainly to display product information, combined with the actual business needs; the interface design scheme can be divided into three categories: one is the basic component class, two is the user-related class, and three is the product-related class. The basic components are the common components of the system. The user-related category mainly involves the interface design of the basic function module, personal center module, student personal center module, and order management module of the system, with user interaction as the focus, aiming to provide a more concise operation mode and a more friendly user experience. The product-related category involves the home page management module, course management module, store management module, and shopping cart management module, aiming to provide richer design elements, a more beautiful style layout, more hierarchical, and clearer theme display effect.

The top part of the personal center page is divided into middle and bottom structures, and the top part is equipped with a website navigation bar, which can locate other pages of the website, such as the home page and shopping cart page, and can quickly log out. The middle part is used to display the current user's personal information, such as name, gender, and address. The bottom part is divided into left and right structures with the largest proportion of pages. The left part is the internal navigation bar of the personal center page, and the right part is the specific function page; when the user clicks on a function in the navigation bar, the right part will jump to its corresponding function page, as shown in Figure 5.

Based on the results, we can summarize the disadvantages of individual differences in the DEAP database: uneven distribution within classes and unbalanced samples. The former relates to the data distribution in the sample space, and the latter relates to the label distribution. It reveals a common phenomenon resulting from the apparent individualization problem in sentiment recognition databases. Traditional inductive learning methods lead to lower prediction performance, so the usual solution is a subject-alone training method based on subjects, while a training process based on all subjects' data does not result in a stable model. Comparison of the results shows that the T-SVR performance using data from all subjects for training is better than the inductive approach based on trainee-alone training, validating the effectiveness of the proposed adaptive sentiment recognition model.

Neighborhood knowledge contributes to the construction of a local classifier that is unaffected by outliers and irrelevant information and can complement the imbalance in data samples from similar remaining subjects. Moreover, the performance of ST-SVR is slightly better than that of T-SVR, which indicates that the proposed method ensures a small prediction error and the effect of sample imbalance is less than that of inductive learning methods even without supplementing the remaining subject data.

DEAP is used as a benchmark database for the methods in this chapter to compare the recognition results under different models. Facing the problem of individualization due to individual differences, the best approach is still based on subject-related training (ST-SVR). However, the application of this approach in practical scenarios is limited. For example, the modal information collected from subjects is derived from short-term events, which cannot cover all possible modal information generated by individuals. Therefore, additional modal information from the rest of the subject sample is needed.

## 4. Discussion

In this study, the SCARED scale was used to assess symptoms in patients with adolescent anxiety disorder, and the results showed a negative correlation between total score and neutral correctness, but there was no impairment in neutral correctness in patients with adolescent anxiety disorder, suggesting that the correctness of responses to neutral stimuli in patients with an adolescent anxiety disorder may be an extrinsic condition causing the severity of anxiety symptoms. An iterative sampling data fusion strategy is also proposed, aiming to integrate and fuse data from multiple sources to make it more effective and further improve the robustness and generalization ability of the model. In the presence of both neutral and negative stimuli, neutral stimuli act as a protective message to protect individuals from negative stimuli, and this study suggests that adolescent anxiety disorder patients show avoidance of neutral stimuli, which may be one of the factors causing the severity of anxiety symptoms, which is consistent with previous studies. Separation anxiety factor scores were negatively correlated with negative accuracy, and social terror factor scores were negatively correlated with negative accuracy and neutral accuracy.

The stimulus materials in this study used emotional faces, and social anxiety was hypothesized to be related to threat-related facial expressions because face information may involve negative evaluations by others, and the point detection paradigm using face pictures was shown to be more specific for separation anxiety, social anxiety, and aversive symptoms in attentional bias based on previous findings, which were verified in this dissertation. In conclusion, avoidance of neutral stimuli may be a risk factor for symptom severity in adolescents with anxiety disorders, and the material used in the paradigm of this study has good sensitivity.

The experimental paradigm design was monotonous, and future studies could be continued to increase the length and number of different stimuli. The follow-up period for the subjects was short, and the follow-up of the postintervention outcomes could not be continued for a long time. This experiment only studied behavioral and symptomatologic aspects, and ERP, eye-tracking technology, and magnetic resonance imaging can be used to further explore related issues in the future. This experiment only focuses on the attentional bias characteristics and interventions of adolescents with anxiety disorders, and the attentional bias characteristics and interventions of adolescents with other mood disorders can be added in the future to further study the attentional bias characteristics and interventions of adolescents with mood disorders.

## 5. Conclusion

After determining the design model and development model, this paper combined the actual business requirements, designed the overall system architecture, determined the design ideas and technology stack for each layer, and presented the functions of each layer of the whole system in the form of diagrams. In addition, this paper lists that each server deployed in the outline design section briefly introduces the functions of each server and shows the system working principle in the form of pictures. The detailed design follows the division and description of the outline design, discusses and designs each functional module of the system in more detail, and implements the corresponding on its basis. This part uses tools such as class diagrams and timing diagrams to provide a detailed description of the relevant details and processes. In addition, the detailed design also specifies the running environment of the system, introduces the design and implementation of the main interfaces, and shows the actual development results through screenshots of the system interface.

## Figures and Tables

**Figure 1:** Valence and arousal degree.

**Figure 2:** Intergroup comparison of the number of children reaching the embodied level by age.

**Figure 3:** System use case role diagram.

**Figure 4:** Semantic analysis results.

**Figure 5:** Detection model test results.

**Table 1:** Differences in emotional understanding ability in terms of gender.

Dimension	Gender	*N*	Mean	Standard deviation
Emotional understanding	Male	72	27.3	50.2
	Female	65	36.4	49
Emotional expression ability	Male	46	45.3	43.8
	Female	61	41.9	27.2
Emotion regulation ability	Male	62	44.5	57.3
	Female	87	21.6	50.6

**Table 2:** Table of product types of educational institutions.

Type	Product sales channels	Product source	How to use the product
Online	This system is sold online	Published by Institutional Headquarters	Online self-study of this system
	79	38	50
	42	87	50
Offline	This system is sold online	Published by Institutional Headquarters	Online self-study of this system
	72	37	54
	69	82	82
Comprehensive	This system is sold online	Published by Institutional Headquarters	Online self-study of this system
	38	37	50
	66	73	79

## Data Availability

The data used to support the findings of this study are available from the corresponding author upon request.
